# Research on the Characteristics of Food Impaction with Tight Proximal Contacts Based on Deep Learning

**DOI:** 10.1155/2021/1000820

**Published:** 2021-11-05

**Authors:** Yitong Cheng, Zhijiang Wang, Yue Shi, Qiaoling Guo, Qian Li, Rui Chai, Feng Wu

**Affiliations:** ^1^Department of Prosthodontics, Shanxi Medical University School and Hospital of Stomatology, China; ^2^Shanxi Provincial Key Laboratory of Biomedical Imaging and Imaging Big Data, College of Big Data, North University of China, China

## Abstract

**Objective:**

Based on deep learning, the characteristics of food impaction with tight proximal contacts were studied to guide the subsequent clinical treatment of occlusal adjustment. At the same time, digital model building, software measurement, and statistical correlation analysis were used to explore the cause of tooth impaction and to provide evidence for clinical treatment.

**Methods:**

Volunteers with (*n* = 250) and without (*n* = 250) tooth impaction were recruited, respectively, to conduct a questionnaire survey. Meanwhile, models were made and perfused by skilled clinical physicians for these patients, and characteristics such as adjacent line length, adjacent surface area, tongue abduction gap angle, buccal abduction gap angle, and occlusal abduction gap angle were measured. A normality test, differential analysis, correlation analysis of pathological characteristics of the impaction group, principal component analysis (PCA), and binary logistic regression analysis were performed.

**Results:**

The adjacent line length, adjacent surface area, tongue abduction gap angle, buccal abduction gap angle, and occlusal abduction gap angle all met normal distribution. There were statistically significant differences in adjacent line length (*p* < 0.001), adjacent surface area (*p* < 0.001), and occlusal abduction gap angle (*p* < 0.001) between the two groups. After dimensionality reduction by PCA on characteristics, adjacent line length, adjacent surface area, buccal abduction gap angle, and occlusal abduction gap angle had a strong correlation with the principal components. Binary logistic regression analysis showed that adjacent line length and adjacent surface area had positive effects on impaction. The buccal abduction gap angle and occlusal abduction gap angle had a significant negative influence on impaction.

**Conclusion:**

Adjacent line length, adjacent surface area, buccal abduction gap angle, and occlusal abduction gap angle are independent factors influencing food impaction.

## 1. Introduction

In daily life, most people have food impaction. During chewing, food impaction occurs when food fragments or fibers wedge into the space between adjacent teeth due to the action of occlusal pressure or gingival retreat, which is called food impaction [1]. According to the different ways of the impaction, impaction can be divided into vertical impaction and horizontal impaction [2]. If it is not clear in time, impacted food will help bacterial reproduction, stimulate adjacent tissue, and cause a series of problems such as periodontal atrophy, gum papillitis, adjacent surface caries, halitosis, heavier periodontitis [3, 4]. As time goes by, oral health problems become more serious [5], which seriously influence people's daily life.

The main causes of occlusal food impaction are [6] caries, occlusal disorder, tooth wear, tooth defect, periodontal disease, alveolar bone atrophy, and other problems [4]. We based on the deep learning theory to study the influence factor for food impaction with tight proximal contacts [6]. We also illustrate problems in the process of food impaction through the analysis of adjacent line length, adjacent surface area, tongue abduction gap angle, buccal abduction gap angle, and occlusal abduction gap angle [7].

In the treatment of food impaction, the cause of the impaction should be identified first, and the treatment should be carried out according to the cause. If there is caries on the adjacent surface, the corresponding filling or repair method should be selected according to the specific situation, and the normal contact relationship should be restored. Restoration treatment should be carried out as soon as possible after tooth loss [8]. Patients with periodontal inflammation should be treated after anti-inflammation [9]. Patients with dental malformations can undergo oral grinding adjustment [10]. As for the treatment of food impaction without anatomical structure destruction, a large number of domestic and foreign literature reports have taken the occlusal adjustment as the basic treatment [3]. It has the advantages of less grinding tissue, easy operation, and easy acceptance by patients. The methods for occlusal adjustment include adjusting the grinding and filling tooth tip, expanding the food overflow channel, deepening the food overflow groove, and adjusting the main functional area of occlusal. According to relevant literature reports, it can be systematically summarized into the following three methods: sequence adjustment [11], adjustment of the main functional area of the bite [12], and measurement of buccal tongue abduction gap angle [13]. The goal of therapy of food impaction with tight proximal contacts is to reshape the close adjacent surface contact [14] and maintain its stability.

Deep learning is a branch of machine learning. It is an algorithm based on the artificial neural network to learn information representation. Deep learning is increasingly widely used in clinical practice. For example, Chung et al. [15] verified the feasibility of automatic segmentation based on deep learning in breast radiotherapy planning. Clinical applications of deep learning include medical image analysis, disease diagnosis, and other aspects [16, 17]. Along with the rapid development of three-dimensional (3D) acquisition technology, 3D data is increasingly applied in the medical field, including the 3D point cloud. Guo and his partners [18] analyzed several deep learning methods for processing 3D point clouds in their study. Based on the LCCP method, Wang et al. [19] segmented the 3D point cloud image of plants based on locally convex connected patches to measure the length, width, and area of leaves. Nevertheless, there is no relevant study using the 3D point cloud network for analysis and processing of tooth characteristic extraction.

Incidence of food impaction with tight proximal contacts is on the rise clinically. In order to improve oral diagnosis and treatment technology and promote the process of treating food impaction with tight proximal contacts, this study is aimed at exploring the characteristics of food impaction with tight proximal contacts [20]. Based on deep learning theory, in recording the steps of tooth segmentation, a comparison method is used to collect and analyze differences of food impaction with tight proximal contacts in adjacent line length, adjacent surface area, tongue abduction gap angle, buccal abduction gap angle, and occlusal abduction gap angle, so as to provide the basis for clinical treatment of adjacency of close food.

## 2. Materials and Methods

### 2.1. Study Object

A total of 500 volunteers (250 for food impaction and 250 for nonfood impaction) who are ages 25 to 50 were recruited according to the eligibility criteria for the study with no gender limitation. Inclusion criteria: (1) dental dentistry was complete, arranged basically neatly, and no adjacent surface caries was found between the first molar and the second molar by clinical examination and X-ray examination; (2) the first molars and the second molars are not loose; and (3) the impaction area between the first molar and the second molar is close, and the measurement of the feeler is less than 60 *μ*m. Exclusion criteria: (1) patients have severe periodontal disease; (2) the impaction is not complete to the jaw; (3) the first or second molars have full crown or inlay restoration or have adjacent surface fillings; (4) there are obvious “steps” between the first molars and the second molars; and (5) between the upper and lower jaws is reverse occlusion, locking occlusion, and other states. The basic information of food impaction was obtained by a questionnaire.

### 2.2. Experimental Materials

The following are the experimental materials: mint and wax dental floss (Qizhimei Commercial and Trading Co., Ltd), DMG Silagum silicone rubber impression material heavy body+light body (DMG Dental, Germany), DMG O-bite Bite record, silicone rubber (DMG dental, Germany), 3-shape TRIOS second-generation oral scanner, silicone rubber blending gun (DMG dental, Germany), and superanhydrite (Heraeus Kulzer).

### 2.3. Experimental Steps

#### 2.3.1. Model Preparation and Perfusion

Oral education was conducted to the volunteers, and the correct way of brushing teeth and using dental floss was instructed. During the process of modeling, subjects should relax and sit and look straight ahead, and the mandibular plane should be parallel to the ground plane. During the detection process, subjects should maintain a constant posture, and those who cannot cooperate well will be excluded. After checking the integrity of the impression, the saliva was cleaned and the dentistry model was injected with superanhydrite by the same molding worker. After demolding, the mold was repaired in accordance with the standard model.

#### 2.3.2. Records of Occlusal Relationship

Volunteers were instructed to clench in the intercuspal position. A silicone rubber Bite record (DMG O-bite Bite record, silicone rubber, Germany) was used to record the posterior occlusal relationship.

#### 2.3.3. Establishment of Digital 3D Scanning Model

A 3-shape scanner was used to scan the repaired upper and lower jaw plaster models and the correct occlusal relationship, and the data in STL format was obtained, as shown in Figure 1.

#### 2.3.4. Deep Learning Network Segment Teeth

Firstly, the tooth STL model was directly transformed into the point cloud model. Due to the excessive number of point clouds and the amount of calculation, the point cloud was subsampled during the network training. Different from the common point cloud preprocessing methods of random sampling and uniform sampling, in order to calculate the tooth impaction characteristics more accurately, and considering the relationship between the tooth impaction characteristics and the tooth surface curvature at the same time, the higher the tooth surface curvature, the higher the probability of containing the tooth impaction characteristics. In this experiment, geometric sampling was used to sample points on the tooth surface. Through variable Deformable Kernel, the location changes of sample points were learned on the basis of rigid sampling.

The segmentation network adopted in this experiment is a segmentation network model provided by the North University of China and constructed based on KPConv [21] kernel convolution. The network model is similar to the U-Net [22] model and consists of two parts, encoder and decoder. It is a symmetric semantic segmentation model. Finally, the segmented point cloud results were mapped to the STL model for visualization, and the teeth were marked with different colors, as shown in Figure 2. Only the first and second molars studied in the experiment were separated to increase the accuracy of network training.

#### 2.3.5. Feature Measurement

The segmented tooth point cloud image was projected horizontally, and then, the teeth were compressed into two-dimensional images to facilitate the measurement of the length of the adjacent line and the fitting of the dividing line. The two farthest points on the dividing line were found as the two ends of the tooth adjacent line; that is, the length of the adjacent line was obtained by measuring the distance between the two ends, as shown in Figure 3.

The tongue and buccal abduction gap angles were measured by horizontal projection based on point cloud images. The two ends of the secant line were extended outward for a fixed length, and a horizontal line was made from the extension line to both sides of the teeth to get the two points nearest to the extension line. The angles composed by the three points were the tongue abduction gap angle and buccal abduction gap angle, as shown in Figure 4.

By projecting the two segmented tooth point cloud images in the vertical direction, the two-dimensional point cloud in the vertical direction of the teeth can be obtained. In accordance with the above method for calculating the tongue abduction gap angle, the occlusal abduction gap angle can be obtained, as shown in Figure 5. At the same time, the tooth partition plane in the vertical direction was taken out to obtain the adjacent surface area, as shown in Figure 6.

### 2.4. Statistical Analysis

Statistical analysis was performed using R software and SPSS 24.0. Kolmogorov-Smirnov and Shapiro-Wilk methods were used to test the normal distribution of the characteristics of the impaction group. An independent sample *T*-test was used to analyze statistical differences in features between the impaction and nonimpaction groups. Correlation analysis was used to test correlations between features. Principal component analysis (PCA) was used for dimensionality reduction of characteristics, and the characteristic value greater than 1 was the screening condition of PCA. Binary logistic regression analysis was used to analyze the effect of characteristics on impaction. *p* < 0.05 was considered statistically significant.

## 3. Results

### 3.1. Normality Test

Normality tests were performed for adjacent line length, adjacent surface area, tongue abduction gap angle, buccal abduction gap angle, and occlusal abduction gap angle in the patients with and without food impaction.  Table 1 displays that the sample size of research data was less than or equal to 50, so the S-W test was used. The results showed that the adjacent line length, adjacent surface area, tongue abduction gap angle, buccal abduction gap angle, and occlusal abduction gap angle all fitted with a normal distribution (*p* > 0.05).

### 3.2. Differential Analysis of Characteristics between the Impaction and Nonimpaction Groups

A *T*-test was used to compare the characteristic differences between the impaction group and the nonimpaction group. The analysis results are shown in Table 2. Statistically significant differences between the two groups were presented in adjacent line length (*p* < 0.001), adjacent surface area (*p* < 0.001), and occlusal abduction gap angle (*p* < 0.001). Additionally, the mean value of the tongue abduction gap angle (*p* = 0.087) and buccal abduction gap angle (*p* = 0.105) in the nonimpaction group was larger than those in the impaction group, but the difference was not statistically significant.

### 3.3. Correlation Analysis of Tooth Characteristics in Food Impaction Patients

It could be seen from Table 3 that the area of the adjacent surface (*ρ* = 0.317, *p* = 0.025) and the length of the adjacent line (*ρ* = 0.297, *p* = 0.036) of food impaction were significantly positively correlated with the tongue abduction gap angle.

### 3.4. PCA

As could be seen from Table 4, for the degree of commonality, there was a total of 1 item involving the tongue abduction gap angle, indicating that the relationship between the principal components and the study item was very weak, and the principal components were unable to effectively extract the information of the study item. Therefore, this item should be deleted and analyzed again after deletion.

After deleting the tongue abduction gap angle data, the main components of the patients with and without impaction were analyzed again. It could be seen from Table 5 that the corresponding communality degree values of all the study items were higher than 0.4, indicating that there was a strong correlation between the study items and the principal components, and the principal components could effectively extract the information. After ensuring that the principal components could extract most of the information of the research item, the corresponding relationship between the principal components and the research item was analyzed (when the absolute value of the loading coefficient was greater than 0.4, it was indicated that the item had a corresponding relationship with the principal components).

### 3.5. Binary Logistic Regression Analysis

The adjacent line length, adjacent surface area, buccal abduction gap angle, and occlusal abduction gap angle were used as independent variables, and the impaction or not was used as the dependent variable for binary logistic regression analysis. The model formula is ln(*p*/1 − *p*) = 0.889∗adjacent line length + 3.396∗adjacent surface area − 0.071∗buccal abduction gap angle − 0.089∗occlusal abduction gap angle − 19.797 (where *p* represents the probability of having impaction and 1 − *p* represents the probability of do not have impaction. Unit: adjacent line length (mm); adjacent surface area (mm^2^); angle (°)).

As displayed in Table 6, the adjacent line length, adjacent surface area, buccal abduction gap angle, and occlusal abduction gap angle had significant effects on the impaction (*p* < 0.05). To be specific, adjacent line length had a positive effect on impaction, and the regression coefficient was 0.889, which passed the significance level test. In other words, if the adjacent line length increased by 1 unit, the probability of impaction increased by 2.432 times. The adjacent surface area also had a positive effect on impaction (regression coefficient = 3.396, *p* < 0.05). Specifically, if the adjacent surface area increased by 1 unit, the probability of impaction increased by 29.835 times. However, the buccal abduction gap angle had a significant negative effect on impaction (regression coefficient = −0.071), which indicated that the probability of impaction decreased by 0.931 times when the buccal abduction gap angle increased by 1 unit. At the same time, the occlusal abduction gap angle had a significant negative effect on impaction (regression coefficient = −0.089), reflecting that the probability of impaction decreased by 0.915 times when the occlusal abduction gap angle increased by 1 unit.

## 4. Discussion

The occurrence of food impaction is usually caused by contact damage of the adjacent teeth, severe abrasion of the occlusal surface, and abnormal contact [23]. This study measured the adjacent line length and adjacent area, tongue abduction gap angle, buccal abduction gap angle, and occlusal abduction gap angle. Statistically significant differences were found in adjacent line length (*p* < 0.001), adjacent surface area (*p* < 0.001), and occlusal abduction gap angle (*p* < 0.001) between the two groups. By increasing the contact surface after occlusal adjustment, the space between adjacent teeth is formed and the food overflow channel is enlarged, which is conducive to food expulsion and alleviating the symptoms of food impaction.

In the process of occlusal adjustment, errors occurred when measuring the tongue abduction gap angle, buccal abduction gap angle, adjacent line length, and so on. By applying a 3-shape scanner, we ensured the accuracy of the data and provided accurate data for occlusal adjustment. The cause of the effect on impaction was determined, the effect of before and after treatment was compared, and a basis for clinical treatment was provided.

The results before and after treatment were compared. According to the above data, when the length of the adjacent line was 3.52 ± 1.62 mm, the area of the adjacent surface was 6.21 ± 2.31 mm^2^, tongue abduction gap angle was 52.24 ± 13.17°, buccal abduction gap angle was 54.15 ± 13.61°, and occlusal abduction gap angle was 89.26 ± 21.64°, the incidence of food impaction decreased.

Wear is the main cause of severe dentition wear [24]. Due to the increased contact area of tooth wear, alveolar bone growth, and mesial displacement of teeth, severe dentition wear may lead to changes in maxillofacial height. This change makes it easy for food to accumulate in the alveolar ridge, forming a lot of small and sharp filled cusps. In the process of transverse transportation of food, it is easy to accumulate on the filled cusps and form a wedge-shaped extrusion, generating an instantaneous mechanical tooth effect on the adjacent surface area.

This study provides a new research method and quantitative standard for the guidance of food impaction with tight proximal contacts. This paper points out a new idea of deep learning and modern information technology in the clinical oral cavity. Through measurement of the tongue abduction gap angle, buccal abduction gap angle, length of adjacent line, and cross-sectional area of the abductive gap channel, we provide a basis for occlusal treatment. These findings will provide new ideas and directions for the treatment of food impaction, guide the formulation of clinical protocols and the choice of treatment methods, and greatly improve the clinical efficacy of food impaction.

However, there are some limitations to this study. Firstly, 250 patients with food impaction were studied and analyzed. Due to the differences in oral symptoms of each patient, there would be some errors in the data analyzed. Secondly, we have studied the main parts that cause food impaction, the first molar and the second molar. Other tooth positions have not been studied, and further improvement is needed in future studies.

In conclusion, deep learning was used to study the characteristics of food impaction with tight proximal contacts. We learned that the main reason affecting food impaction with tight proximal contacts was the close relationship between the adjacent surface contact area of adjacent teeth. Our results will provide a new research direction for the clinical treatment of food impaction and guide the treatment of food impaction with tight proximal contacts to improve the symptoms of food impaction.

## Figures and Tables

**Figure 1:** 3D model data obtained after scanning: (a) maxillary 3D model data; (b) mandibular 3D model data; (c) left occlusal relationship; (d) right occlusal relationship.

**Figure 2:** Point cloud of first molars and second molars.

**Figure 3:** The length of adjacent lines measured by horizontal projection.

**Figure 4:** The tongue abduction gap angle and buccal abduction gap angle measured by horizontal projection.

**Figure 5:** The angle of the spread gap measured by vertical projection.

**Figure 6:** The area obtained by cutting the plane.

**Table 1:** Result of normality test.

Item	Sample size	Mean value	Standard deviation	Skewness	Kurtosis	Kolmogorov-Smirnov test		Shapiro-Wilk test	
						*D* value	*p* value	*W* value	*p* value
Adjacent line length	500	4.272	0.959	0.074	0.396	0.108	0.157	0.978	0.476
Adjacent surface area	500	8.290	0.394	0.275	0.306	0.128	0.040^∗^	0.977	0.423
Tongue abduction gap angle	500	50.246	9.882	0.236	0.049	0.058	0.941	0.990	0.947
Buccal abduction gap angle	500	50.983	11.797	0.312	1.067	0.069	0.793	0.972	0.267
Occlusal abduction gap angle	500	58.916	29.429	0.235	-0.280	0.084	0.516	0.973	0.317

Note: ^∗^*p* < 0.05.

**Table 2:** *T*-test for characteristics of impaction and nonimpaction patients.

Characteristics (mean (SD))	Nonimpaction	Impaction	*p* value
Adjacent line length	3.304 (1.187)	4.267 (0.937)	<0.001
Adjacent surface area	7.763 (0.466)	8.278 (0.390)	<0.001
Tongue abduction gap angle	53.630 (10.275)	50.236 (9.673)	0.087
Buccal abduction gap angle	55.849 (15.047)	51.462 (12.121)	0.105
Occlusal abduction gap angle	92.006 (13.091)	59.466 (29.288)	<0.001

Note: ^∗^*p* < 0.05.

**Table 3:** Correlation analysis of tooth characteristics in food impaction patients.

		Adjacent surface area	Adjacent line length
Tongue abduction gap angle	Correlation coefficient	0.317	0.297
	*p* value	0.025^∗^	0.036^∗^
Buccal abduction gap angle	Correlation coefficient	0.077	0.171
	*p* value	0.594	0.236
Occlusal abduction gap angle	Correlation coefficient	0.078	0.036
	*p* value	0.592	0.803

Note: ^∗^*p* < 0.05; ^∗∗^*p* < 0.01.

**Table 4:** Principal component analysis of impaction and nonimpaction.

Item	Loading coefficient		Communality (common factor variance)
	Principal component 1	Principal component 2	
Adjacent line length	**0.707**	0.111	0.513
Adjacent surface area	**0.719**	0.069	0.522
Tongue abduction gap angle	0.051	**0.596**	0.358
Buccal abduction gap angle	-0.168	**-0.757**	0.601
Occlusal abduction gap angle	**-0.650**	**0.439**	0.615

Note: the numbers in the table are overstriking: bold means the absolute loading factor coefficient is greater than 0.4; otherwise is less than 0.4.

**Table 5:** Principal component analysis of impaction and nonimpaction (adjusted).

Item	Loading coefficient		Communality (common factor variance)
	Principal component 1	Principal component 2	
Adjacent line length	**0.705**	-0.100	0.507
Adjacent surface area	**0.719**	-0.134	0.535
Buccal abduction gap angle	-0.158	**0.909**	0.851
Occlusal abduction gap angle	**-0.657**	**-0.472**	0.654

Note: the numbers in the table are overstriking: bold means the absolute loading factor coefficient is greater than 0.4; otherwise is less than 0.4.

**Table 6:** Results of binary logistic regression analysis were summarized.

	Regression coefficient	Standard error	Wald *χ*^2^	*p*	OR	OR value 95% CI	
						Lower limit	Upper limit
Adjacent line length	0.889	0.333	7.108	0.008	2.432	1.265	4.676
Adjacent surface area	3.396	0.933	13.240	<0.001	29.835	4.790	185.819
Buccal abduction gap angle	-0.071	0.031	5.119	0.024	0.931	0.876	0.991
Occlusal abduction gap angle	-0.089	0.022	16.310	<0.001	0.915	0.877	0.955

## Data Availability

The data that support the findings of this study are available on request from the corresponding author. The data are not publicly available due to privacy or ethical restrictions.
